# The Emerging Role of Nanomedicine in the Management of Nonalcoholic Fatty Liver Disease: A State-of-the-Art Review

**DOI:** 10.1155/2021/4041415

**Published:** 2021-10-08

**Authors:** Seyedeh Alia Moosavian, Thozhukat Sathyapalan, Tannaz Jamialahmadi, Amirhossein Sahebkar

**Affiliations:** ^1^Nanotechnology Research Center, Pharmaceutical Technology Institute, Mashhad University of Medical Sciences, Mashhad, Iran; ^2^Department of Academic Diabetes, Endocrinology and Metabolism, Hull York Medical School, University of Hull, Hull HU3 2JZ, UK; ^3^Department of Nutrition, Faculty of Medicine, Mashhad University of Medical Sciences, Mashhad, Iran; ^4^Biotechnology Research Center, Pharmaceutical Technology Institute, Mashhad University of Medical Sciences, Mashhad, Iran; ^5^Applied Biomedical Research Center, Mashhad University of Medical Sciences, Mashhad, Iran; ^6^School of Pharmacy, Mashhad University of Medical Sciences, Mashhad, Iran

## Abstract

Nonalcoholic fatty liver disease (NAFLD) is a common chronic liver disease that can lead to end-stage liver disease needing a liver transplant. Many pharmacological approaches are used to reduce the disease progression in NAFLD. However, current strategies remain ineffective to reverse the progression of NAFLD completely. Employing nanoparticles as a drug delivery system has demonstrated significant potential for improving the bioavailability of drugs in the treatment of NAFLD. Various types of nanoparticles are exploited in this regard for the management of NAFLD. In this review, we cover the current therapeutic approaches to manage NAFLD and provide a review of recent up-to-date advances in the uses of nanoparticles for the treatment of NAFLD.

## 1. Introduction

Nonalcoholic fatty liver disease (NAFLD) is the deposition of fat (steatosis) in the liver, excluding the secondary causes of fatty liver, such as excessive alcohol consumption, viral hepatitis, or certain medications. NAFLD is commonly associated with metabolic syndromes such as obesity, hypertension, diabetes, hyperlipidemia, and hypertriglyceridemia. Studies have shown that NAFLD-related liver diseases are escalating as a public health issue. Because of the increasing prevalence of obesity and type 2 diabetes worldwide, NAFLD is emerging as the critical risk factor for end-stage liver disease and liver cancer. NAFLD is expected to become one of the most common indications for liver transplantation in the next decade [1–4].

NAFLD encompasses a spectrum of liver abnormalities. Various histological grades have been described in the evaluation of NAFLD, including simple steatosis (grade 1), steatosis with lobular inflammation and ballooned hepatocytes (grade 2), and lobular inflammation, ballooned hepatocytes, and fibrosis (grade 3). NAFLD can progress to cirrhosis, hepatocellular carcinoma, and liver failure [5, 6].

### 1.1. Pathogenesis of NAFLD

Multiple factors are involved in the pathogenesis of NAFLD [7]. Genes, hormones, and nutrition can contribute to the development of NAFLD. It is well established that hepatic fat accumulation is related to insulin resistance, leading to steatosis development [8].

The pathophysiology of NAFLD and its development is a complex process with many unsolved topics. One prevailing model for describing the pathogenesis of NAFLD and NASH (nonalcoholic steatohepatitis) is the “two-hit hypothesis.” Triglyceride accumulation in the liver is attributed as the first hit. The second hit which can make NAFLD progress to severe liver injuries is mediated by several factors, including oxidative stress, cytokines, and mitochondrial dysfunction [9, 10].

The original “two-hit” approach cannot fully explain the pathophysiology of NAFLD, which incorporates several variables. Many studies in recent decades have revealed that the gut microbiota plays an essential role in NAFLD development via the gut-liver axis (GLA). Furthermore, significant progress has been made in the previous decade, with the involvement of inflammation and high-sugar diets emerging as key players in the etiology of NAFLD. With the advancement of technology, more researchers have focused on genetic predispositions and discovered several gene variations that may modify lipid and sugar metabolism in the liver and other tissues, such as adipose tissue (Figure 1) [10, 11].

### 1.2. Management of NAFLD

There is no available effective pharmacotherapy to prevent the progression of NAFLD to NASH and advanced stages of hepatic fibrosis and cirrhosis [12]. Because of the complexity of NAFLD pathophysiology, different severity levels of disease, and the heterogeneity of the patient population, developing a drug for the treatment of NAFLD is challenging [13]. Some anticipated efficient drugs have been failed in the last stages of clinical trials [14]. Current therapeutic approaches to NAFLD include lifestyle changes and diet, associated metabolic disorders, lipid-lowering agents, and insulin-sensitizing medications to reduce weight. In addition, natural compounds and antioxidant supplements have been studied to reduce the NAFLD symptoms. The major drawback of pharmacotherapy in liver diseases is the inability to achieve therapeutic concentration in the hepatic tissue. Additionally, targeting drugs to specific cells in liver tissue can be challenging [8].

Nanoparticles (NPs) as drug carriers have shown to have tremendous potential for the management of NAFLD. Nanoparticles offer great promise in improving the bioavailability of drugs due to their size and surface characteristics, protection of drugs from degradation, increasing gastrointestinal absorption, and increasing cellular uptake at the target site. In addition, NPs are designed to accumulate in the desired tissue such as the liver, reduce the clearance of the drug, reduce drug accumulation tissues other than the liver, and increase the cell-specific uptake of the liver. Thus, a wide range of NPs has been designed for targeted drug delivery to the liver.

Employing NPs for liver drug delivery has been discussed in previous reviews [15–18]. This review covers the current therapeutic approaches to manage NAFLD and provides a review of recent advances in the uses of nanoparticles to treat NAFLD.

### 1.3. Liver Targeting of Nanoparticles

The liver comprises hepatocytes, Kupffer cells, and fenestrated endothelial cells (Figure 2). Kupffer cells, the liver's resident macrophage population, are known to phagocytose foreign particulates. Most of the nanoparticles are typically taken up by Kupffer cells in the liver, which preferentially interact with negatively charged NPs. Kupffer cells are responsible for immune and inflammatory responses and regulate liver diseases, including NAFLD. Hepatocytes, which are specialized epithelial cells, also interact with NPs but to a lower extent than the macrophages. They activate other liver cells and are also involved in immune and inflammatory responses. In contrary to Kupffer cells, hepatocyte uptake of NPs increases with positive zeta potential. Liver sinusoidal endothelial cells (LSECs) are specialized endothelial cells that form the interface between blood cells and liver cells. Open fenestrations and lack of basal lamina of LSECs provide a mesh-like structure leading to the entrapment of NPs in the liver. Stellate cells are fat-storing cells that play a crucial role in liver fibrosis [17, 19].

### 1.4. Passive Targeting

Passive targeting refers to a preferential accumulation of NPs in the liver. This preferential distribution to the liver is attributed to the presence of fenestrations along the endothelial barrier of the liver and the absence of basal lamina. After systemic administration, the majority of NPs with a size above 6 nm accumulate in the liver. Thus, enterohepatic circulation plays a vital role to deliver orally administered NPs to the liver [20].

Nonparenchymal cells located at the sinusoidal endothelium (i.e., Kupffer cells) are responsible for passive targeting due to their location in the liver sinusoid. Nanoparticles with the size of >100 nm mostly accumulate in sinusoidal endothelial cells and Kupffer cells, while the smaller nanoparticles (<100 nm) passively target hepatocytes and hepatic stellate cells [21]. The optimum size of NPs for liver delivery is about 40–150 nm [22].

### 1.5. Active Targeting

Most NPs, after intravenous injection, spontaneously accumulate in the liver by the action of RES. In passive targeting, NPs accumulate in Kupffer cells which are resident liver macrophages. If the destination is other liver cells, PEGylation and active targeting are appropriate strategies. PEGylation is the general strategy to inhibit opsonization in plasma and consequently reduce nonspecific entrapment by macrophages [23].

Active targeting involves employing affinity ligands on the surface of NPs for specific uptake by the targeted liver cells. As mentioned before, the liver comprises different cell types with various specific activities. These cells express various ligands which have different pathological significances (Figure 3). Active targeting is a promising way to deliver nanoparticles to a specific population of liver cells. Many ligand-targeted approaches have been explored in the management of liver diseases. The hepatocytes are the main target of treatment in NAFLD. To achieve high therapeutic efficiency, specific targeting to hepatocytes is essential. The design of actively targeted NP drug carriers for liver cells is complex because different cells express receptors with similar functions. The ligands that can be used for receptor-mediated delivery systems are presented in Figure 3.

### 1.6. NPs for the Treatment of NAFLD

To date, different NPs have been employed as drug delivery systems to enhance treatment response in NAFLD. Various research studies on the liver targeting NPs used in the treatment of NAFLD are reviewed below.

### 1.7. Nanoemulsions

Nanoemulsions (NEs) are very fine oil-in-water dispersions in which the size of droplets ranges from 50 to 500 nm [24]. Because of their thermodynamic stability, they offer exciting properties compared to conventional emulsions. NEs are more stable over time. They have a transparent appearance and also control drug release rate and target specificity. Al-Okbi et al. formulated pumpkin seed oil in NEs and showed their oral administration improves dyslipidemia, oxidative stress, and liver dysfunction observed in rats. However, they did not use conventional formulation to compare the results [25].

Vitamin D is a fat-soluble vitamin that has a wide range of functions in the body. Many studies have shown the beneficial roles of vitamin D supplements in managing NAFLD [26–29]. However, the role of vitamin D supplementation in NAFLD is still controversial [16–21]. Encapsulation of vitamin D in nanoparticles has been investigated to improve the stability and bioavailability of this vitamin in several studies, while some studies assessed the anti-inflammatory and antioxidant activity of vitamin D. El-Sherbiny et al. compared the bioavailability, solubility, and chemical stability of vitamin D NEs with conventional formulations. They prepared pea protein NEs and reported vitamin D NEs to display better efficiency than the current commercial formulation in rats [30].

Cuminaldehyde is a natural aldehyde organic compound that has antidiabetic and anticancer activities. Haque and Ansari investigated the hepatoprotective effect of cuminaldehyde in rats [31]. Recently, Adu-Frimpong et al. showed formulation of cuminaldehyde in self-emulsified NEs and improved its bioavailability in a rat model. They also evaluated the anti-inflammatory, antioxidative, and antihepatotoxic effects of cuminaldehyde NEs in Kunming mice. They reported that cuminaldehyde NEs reduced the levels of tumour necrosis factor-alpha and interleukin-6, while aspartate aminotransferase, alanine aminotransferase, and malonaldehyde levels were significantly decreased [32].

Silymarin is a polyphenolic flavonoid derived from the purified extract of seeds and fruits of *Silybum marianum*. It is used in chronic liver diseases because of its antioxidant and anti-inflammatory effects [33]. Because of its low water solubility, the oral bioavailability of silymarin is very low. Various nanoparticle delivery platforms were formulated to improve the gastrointestinal (GI) absorption and oral bioavailability of silymarin. The results of these studies have been comprehensively reviewed before [34, 35]. Ahmed et al. encapsulated silymarin in NEs by the aqueous titration method. The oil phase was composed of Sefsol 218 (5.8% v/v), Kolliphor RH40, and polyethylene glycol 400 (S_mix_; 2 : 1; 28.99% v/v). Their results suggest that silymarin NEs could improve the hepatoprotective efficiency of silymarin [36] Yang et al. formulated silymarin NEs employing the spray-drying method. They showed that the silymarin oral bioavailability was about 1.3-fold higher than the commercial product (Legalon^®^) [37].

Calligaris et al. investigated the effect of oil type on silymarin solubility, in vitro bioavailability, and stability. The results indicated that in vitro bioaccessibility of silymarin was not affected by the oil type. In contrast, the oil type affected the nanoemulsion particle size, affecting the stability during the storage. NEs containing extravirgin oil and sunflower oil had less stability than castor oil NEs [38]. Nagi and coworkers prepared silymarin NEs using the high-pressure homogenization (HPH) technique. The droplet size was about 50.02 ± 4.5 nm. The pharmacokinetic studies in rats showed NEs enhanced oral bioavailability compared with silymarin suspension [39].

Carotenoids are lipid-soluble pigments, which can be found in many kinds of fruits and vegetables [40]. Lutein is an oxygenated carotenoid that has potential antioxidant and anti-inflammatory effects. The efficiency of lutein in the treatment of NAFLD has been investigated in several studies [41–43]. However, the oral bioavailability of lutein is poor. It depends on too many factors such as the composition of foods, amount of dietary fat, and food processing such as homogenization or heat treatment [44]. Murillo et al. compared the bioavailability of NE lutein and powdered form in guinea pigs. The results indicated that higher plasma concentration was obtained with NEs [43].

### 1.8. Liposomes

Liposomes are spherical lipid bilayers enclosing an aqueous core that can carry either hydrophilic or hydrophobic drugs [45]. Since the discovery by Bangham in the 1960s, liposomes have been used in different ways as drug vehicles [46]. Owing to several advantages of liposomes, including biocompatibility, biodegradability, and the ability to carry a large payload, liposomes have been employed as a carrier of numerous molecules [47].

In 2016, Cao et al. prepared fenofibrate nanoliposomes and evaluated their inhibitory effects on NAFLD in mice. Liposomes were prepared with soybean lecithin and cholesterol using the dry-film dispersing method. The results showed that treatment with liposomal formulation increases fenofibrate plasma concentration and reduces excessive hepatic lipid significantly. The authors suggested that fenofibrate nanoliposomes could also be efficient in preventing and treating NAFLD [48]. In the same study, the authors found that liposomal formulation significantly improved oral absorption of naringenin and improved hepatoprotective effects on NAFLD [49]. Naringenin is a flavonoid aglycone with many potential biological effects that has a very short half-life (only 30 S) and poor bioavailability [50]. Anti-inflammatory, antitumor, antimicrobial, antiviral, and hepatoprotective effects of naringenin have been widely studied [51]. The results of many studies have shown that encapsulation in nanoparticles could improve the stability, solubility, and bioavailability of naringenin [52].

Chen et al. prepared liposomes containing bile salts to improve fenofibrate bioavailability. They prepared liposomes composed of soybean phosphatidylcholine (SPC) and sodium deoxycholate (SDC) using the dry-film dispersing method followed by sonication and homogenization. Their results showed that bioavailability of fenofibrate increased in rats after oral administration incorporated in liposomes [53].

Baicalin is a flavonoid that has been shown to have hepatoprotective and anti-inflammatory effects. In a study, baicalin-encapsulated nanoliposomes were found to be more effective than free baicalin. Encapsulation in liposomes improves the bioavailability of baicalin and effectively protects mice against MCD-induced NAFLD [54]. Deoxyschizandrin (DS) is a lignin that is found in the fruit of *Schisandra chinensis*. Many studies have confirmed the effect of detoxifying activity and inhibition on adipocyte differentiation of DS [55, 56].

Liu et al. tried to improve the bioavailability of DS by liposomal formulation. Their findings suggest that DS liposomes can alleviate the effects of NAFLD more efficiently than DS solution [54]. Chang et al. studied the hepatoprotective effect of liposomal eicosapentaenoic acid (EPA) and docosahexaenoic acid (DHA). The EPA and DHA liposomes reduced the serum AST and ALT levels and ameliorated NAFLD [57].

Curcumin is a polyphenol with a myriad of biological effects, including antioxidant and anti-inflammatory activities [58–62]. Despite numerous therapeutic potentials, low oral bioavailability has been suggested as a factor limiting its clinical efficacy. The hepatoprotective effect of curcumin has been widely studied before. However, its beneficial effects are limited due to the poor absorption efficacy. Employing nanocarriers such as liposomes, microspheres, emulsions, and micelles has been investigated as a promising strategy to enhance the bioavailability of curcumin [63–65].

Employing a passive targeting mechanism, Maradana et al. used liposomal curcumin to target hepatic myeloid cells. Since hepatic macrophages play an essential role in hepatic diseases such as NAFLD and NASH, immunomodulatory compounds can treat these conditions. The results showed that liposomal curcumin could suppress hepatic inflammation and reduce fat accumulation [66].

Self-emulsifying drug delivery systems (SEDDS) are defined as a mixture of oil, solvent, surfactant, and cosurfactant that can be used for oral delivery of highly lipophilic drugs. After the dispersion of SEDDS in gastrointestinal fluids, micro- or nanoemulsions containing the solubilized drug are yielded that can improve the oral bioavailability of poorly water-soluble drugs [67]. For example, SEDDS have been employed to enhance the oral absorption of silymarin in several studies.

In a study, silymarin was encapsulated in a lipid-based self-microemulsifying drug delivery system (SMEDDS). The pharmacokinetic profile of this preparation was compared with silymarin suspension and solution in rabbits. The formulation consisted of silymarin, Tween 80, ethyl alcohol, and ethyl linoleate. The results showed the bioavailability of SMEDDS was significantly higher than other formulations. The authors suggested the lymphatic transport pathway could have improved the absorption of SMEDDS [68]. In the same study, Li et al. developed SMEDDS using Cremophor EL, ethyl alcohol, ethyl linoleate, and silymarin. The results indicated that the oral bioavailability of silymarin SMEDDS was 2.2-fold higher than the commercial silymarin preparation hard capsule (Legalon^®^) in dogs [69].

In the same study, Wei et al. formulated silybin in a supersaturated self-emulsifying drug delivery system (S-SEDDS) to improve its bioavailability. Labrafac^®^ CC was used as oil phase, while Cremophor^®^ RH 40, Transcutol^®^, and Labrasol^®^ were all used as surfactant and cosurfactant, respectively. The droplet size of S-SEDDS is smaller than conventional SEDDS; hence, it improved the bioavailability of silybin significantly [70].

Woo et al. prepared a silymarin SEDDS using 10% GMO as the oil phase and 15% SLM. In addition, the mixture of Tween 20 and HCO-50 was used as surfactant and Transcutol^®^ was added as cosurfactant. They showed that, in an aqueous medium, the nanoemulsion yielded with the mean droplet size of the internal oil phase of 67 nm. Their results also showed that oral bioavailability of SEDDS was significantly higher compared to commercial silymarin [71].

### 1.9. Micelles

As a colloidal suspension, micelles have been proven as promising drug carriers due to their small particle size, excellent stability, reproducible scale-up, and wide drug loading range [72–75]. Surveying the literature reveals that different micelles have been employed as potential liver drug delivery systems [76]. Mahli et al. investigated the efficiency of micellar solubilization to enhance poor oral bioavailability of xanthohumol. They found that their micellar solubilization xanthohumol had higher bioavailability than native xanthohumol extract and reduced the required dose accordingly. The micellar xanthohumol efficiently inhibited the hepatic steatosis in the Western-type diet (WTD) induced model of inflammation and fibrosis in the C57BL/6 mice model [77]. SKLB023 is a novel 5-benzylidenethiazolidine-2,4-dione derivative that inhibits inducible nitric oxide synthase and, therefore, can reduce nonalcoholic steatohepatitis (NASH) progression. Li et al. encapsulated SKLB023 into phosphatidylcholine-bile salt-mixed micelles to enhance its water solubility and bioavailability. They studied the effect of micellar SKLB023 on activated rat hepatic stellate (HSC-T6) cells since their activation and proliferation are an important factor in the progression of NASH-related liver fibrosis. The results indicated that water solubility of SKLB023 increased 300-fold and micellar formulation significantly inhibited proliferation of HSC-T6 cells compared with free SKLB023. Furthermore, micellar SKLB023 alleviated hepatic lipid accumulation, inflammation, and fibrosis significantly greater than free SKLB023 in the mice model [78].

Resveratrol is a nonflavonoid polyphenol found in numerous plant species. The antioxidant and anti-inflammatory effects of resveratrol have been demonstrated in numerous studies [79] though clinical efficacy has also been argued [80, 81]. The efficacy of resveratrol in treating different liver diseases has been comprehensively reviewed by Izzo and coworkers [82]. Despite the potential benefits, the oral bioavailability of resveratrol is very low. Following oral administration, resveratrol undergoes rapid and extensive metabolism in the intestine and liver. Encapsulation in nanoparticles is an efficient approach to improve the bioavailability of resveratrol [83, 84].

Izdebska et al. investigated the beneficial effect of resveratrol on steatosis in hepatocytes. Their findings showed that resveratrol inhibited oleic acid/palmitic acid-induced steatosis in HepG2 cells and reduced oxidative stress [85]. In another study, they showed resveratrol reduced the glucose-induced steatosis in HepG2 cells and increased the mitochondrial activity of cells [86]. However, in both studies, resveratrol did not affect the viability of HepG2 cells.

Teng et al. prepared an active targeted resveratrol delivery system using lysozyme micelles coated with D-(+)-galactose (Gal) conjugated oxidized starch (Gal-OS) polymer. They partially hydrolyzed lysozymes and prepared micelles using lysozyme peptides. They demonstrated that this targeted resveratrol NPs could effectively reduce hepatic lipid accumulation and insulin resistance and ameliorate NAFLD [87].

### 1.10. Polymeric Nanoparticles

Polymeric NPs are tailor-made NP drug delivery systems that offer many advantages, such as improved bioavailability and selective delivery of drugs to their target tissues [88]. Poly(D,L-lactide-co-glycolide) (PLGA) is a biodegradable and biocompatible polymer that FDA approves for biomedical applications in humans [79]. In a series of double-blind, randomized, placebo-controlled clinical trials, Jazayeri-Tehrani et al. showed PLGA-nanoparticle loaded curcumin reduces inflammatory factors, nesfatin, and appetite in obese patients with NAFLD [89–91]. Wan et al. prepared resveratrol-loaded PLGA nanoparticles by the oil/water (O/W) emulsion technique. Prepared nanoparticles had remarkable encapsulation efficiency (EE%) (97.25%), were also stable enough to be stored at 4°C for at least six months, and reduced hepatocellular proliferation more compared to free resveratrol [92]. Zhao et al. incorporated rapamycin in mPEG-PLGA nanoparticles. They prepared nanoparticles using an emulsion/solvent evaporation method. The therapeutic efficacy of formulations was studied on oleic acid/palmitic acid-induced steatosis in HepG2 cells and the livers of mice with NAFLD induced by a high-fat diet (HFD). Their findings showed rapamycin NPs significantly ameliorate NAFLD in the mice model compared with free rapamycin [93].

Bisindolylmaleimide I (BIM-I) is a protein kinase C inhibitor with anti-inflammatory and antimetastatic properties. Despite the therapeutic potential of BIM-I in the treatment of inflammatory liver diseases, its efficiency has been limited by its poor water solubility and severe side effects. Shkodra-Pula et al. encapsulated BIM-I in PLGA NPs to enhance its bioavailability [88]. Recently, the same group targeted PLGA-encapsulated BIM-I NPs with the near-infrared dye DY-635 for selective delivery of NPs to hepatocytes. Their results showed that active targeting by DY-635 improved in vivo cellular uptake of PLGA-encapsulated BIM-I NPs [94].

Polyurethane (PU) NPs are promising drug delivery systems due to their suitable mechanical properties and biocompatibility [95]. Cao et al. investigated the efficiency of polyurethane nanoparticle-loaded fenofibrate in the treatment of NAFLD. The results indicated that polyurethane-fenofibrate nanoparticles improved the pharmacokinetic profile of fenofibrate and therefore enhanced the inhibitory effects of FNB on NAFLD [96]. Sasaki et al. developed a colloidal nanoparticle dispersion of curcumin (theracurmin) that increases the bioavailability of curcumin 40-fold higher than curcumin powder. They dispersed curcumin in the gum ghatti solution and used a high-pressure homogenizer to optimize dispersion size [97]. Yang et al. investigated the effectiveness of theracurmin in preventing NAFLD in mice models. Theracurmin treatment lowered hepatic triglyceride and total cholesterol levels and significantly reduced lipid peroxidation. Their findings revealed that theracurmin has the potential to control lipid metabolism and can prevent NAFLD [98]. Liu et al. formulated novel PEGylated curcumin with mPEG454 and showed that it significantly reduced hepatic lipid accumulation in high-fat diet (HFD) induced NAFLD mice [99].

Kupffer cells (KCs) are liver-resident macrophages. KC activation is responsible for liver injuries such as NAFLD [100]. Therefore, one strategy to treat liver diseases is the modulation of KC functions. Canup et al. employed PEI-CD98 siRNA-loaded PLAcore/PVAshell to reduce CD98 marker, a factor that is overexpressed in NAFLD, in a mice model. The intravenous administration of CD98siRNA NPs effectively targeted KCs, leading to a significant decrease of major proinflammatory cytokines and markers [101]. Targeting strategies of hepatic macrophages using different nanoparticles was comprehensively reviewed by Colino and colleagues [100].

### 1.11. Nanogels

Nanogels are highly cross-linked polymeric particles that can swell in biological fluids and controlled release their payload. More recently, Mauri et al. encapsulated hydroxytyrosol (HT), a natural polyphenol, in polyethylene glycol and polyethyleneimine based nanogel and evaluated its hepatoprotective effect in vitro. Their results showed that HT-loaded nanogels significantly decrease intracellular triglycerides without induction of oxidative stress in cells [102].

### 1.12. Inorganic Nanoparticles

Cerium oxide nanoparticles (CeO2NPs) possess hepatoprotective potential due to their antioxidant properties. In a study, the antilipogenic effect of CeO2NPs was investigated for the treatment of NAFLD. The results indicated treatment with CeO2NPs alleviated the liver fat accumulation and reduced the expression of genes involved in inflammation. These findings suggest that CeO2NPs could have enormous potential in the treatment of NAFLD [103]. These findings were in line with Oro et al. study that showed CeO2NP administration to CCl4-treated rats reduces steatosis and portal hypertension and the intensity of the inflammatory response [104]. Recently, Carvajal et al. also reported that CeO2NPs protect hepatocytes from cell-induced oxidative damage, reduce the expression of genes involved in inflammation, and regulate kinase-driven cell survival pathways [105]. At the same time, Parra-Robert and colleagues investigated the cellular mechanism of CeO2NPs. They used HepG2 cells as an in vitro model of hepatocellular steatosis. Their results showed that CeO2NPs directly reduced oxidative stress and fatty acid content in steatotic conditions by changes in fatty acid metabolism [106].

### 1.13. Zinc Oxide Nanoparticles

ZnO-NPs are promising novel particles with a wide variety of applications [107]. Sharma et al. showed ZnO-NPs could induce apoptosis in macrophages by modulation of their energy state [108]. Dogra et al. studied the effect of ZnO-NPs on reducing hepatic steatosis by taking advantage of ZnO-NPs on macrophages. The efficiency of ZnO-NPs in the treatment of NAFLD was studied in a mice model. Their experiments using western blot analysis, SiRNA transfection, and immunohistochemistry demonstrated the protective mechanism of ZnO-NPs. Their observations also indicated ZnO-NPs significantly decreased HFD-induced hepatic steatosis and insulin resistance in the mice model [109].

### 1.14. Other NPs

Some studies have determined various microRNAs involved in the development of liver diseases such as NAFLD [110–114]. He et al. found that microRNA-146b (miR-146b) plays an important role in the occurrence and development of NAFLD. They used lactosylated poly(2-dimethylaminoethyl methacrylate) (Lac-PDMAEMA) to target miR-146b mimic delivery to hepatic cells in NAFLD mice. In addition, they evaluated the inhibitory effects of miR-146b mimic in a NAFLD mouse model. Their results showed that Lac-PDMAEMA/miR-146b mimic inhibits fat accumulation in hepatocytes in vitro and effectively alleviates hepatic steatosis in NAFLD mice [115].

Interleukin-22 (IL-22) is a member of the IL-10-like cytokine family. Studies have shown that IL-22 plays an important role in controlling NAFLD and other metabolic diseases. Zai et al. used penetratin-based hybrid nanoparticles to exert liver-targeted IL-22 gene delivery. They constructed metformin-chitosan and showed that this hybrid nanoparticle exerted liver-targeted IL-22 gene delivery and has the potential ability to treat NAFLD. They claimed that since metformin has potential therapeutic benefits for NAFLD in both experimental and clinical studies, metformin-modified chitosan (CM) could be a promising gene delivery platform for NAFLD [116].

In a study, Rafique et al. investigated the efficiency of PEGylated lipid nanoparticles with the core of triolein-POPC (2-oleoyl-1-palmitoyl-*sn*-glycero-3-phosphocholine) in the improvement of pharmacokinetic profile and macrophage accumulation of calcitriol. Their findings showed that calcitriol could be effectively targeted to macrophages using lipid nanoparticles [117].

Nanocrystals (NCs) are stable submicron drug particles (10–1000 nm) that can overcome the solubility difficulties of various drugs. Compared to other nanoparticles, NCs have the simplest composition, more efficient particle size, and higher drug loading. For example, Singh et al. showed that trans-resveratrol (t-RES) NCs represent promising results to improve the oral bioavailability of resveratrol [118].

Albumin is a blood plasma protein produced by hepatocytes. Albumin is a multifunctional protein that has been widely studied as a drug carrier due to its biodegradability, nontoxicity, and nonimmunogenicity [119]. Huang and colleagues demonstrated that galactosylated albumin nanoparticles (Gal-BSA NPs) could improve the oral bioavailability of curcumin through the double absorption mechanisms of passive and active transport. Furthermore, employing a potential strategy of targeted albumin NPs may achieve higher-efficiency intestinal absorption [120].

### 1.15. Challenges in Designing Nanoparticles for Clinical Applications

Despite advances being achieved by NP delivery systems, there are still many obstacles to overcome to utilise the benefits fully. Many articles have comprehensively discussed the challenges in NP drug delivery systems [16, 17, 23]. This is in part associated with the scale-up and commercialization issues, expensive and time-consuming production process, and translating animal studies to clinical trials in humans.

Toxicity associated with NPs should be considered, especially for inorganic nanoparticles [16, 121]. NPs for the treatment of NAFLD also encounter unique barriers as compared with other diseases. Because of the specific physiological function of the liver, NPs accumulate in the liver after administration without any targeting strategy, and therefore, employing nanocarriers would be a simple and promising way to enhance the efficiency of liver disease treatment, while most NPs may not accumulate in the target cells in liver tissue. We require the rational design of NPs, based upon the mechanism of encapsulated medicine and understanding the interaction between NPs and liver cells in vivo. Since the accumulation of NPs in the liver may result in inflammation, exploiting biodegradable and biocompatible NPs for liver delivery is crucial.

Intravenous administration was reported as the most effective route to target NP-encapsulated drugs into the liver efficiently. Intravenously administrated NPs have been shown to work perfectly in *in vitro* and animal studies. However, they do not show significant effects in clinical trials. One possible reason is recognition by the immune system that affects the biological identity of nanoparticles and triggers immunological side effects in clinical trials.

The size of intravenously administrated NPs should be optimized to achieve an appropriate half-life. Decorating NPs by biologically inert hydrophilic polymers, such as PEG, is a promising approach to reduce opsonization by blood proteins and reducing immunogenicity. PEGylation also prevents the agglomeration of NPs and prolongs their shelf-life [17]. Oral delivery is a convenient way of drug administration in the treatment of liver disease. However, because of several natural biological barriers in the gastrointestinal tract, the bioavailability of many drugs reduces after oral administration. Low solubility and permeability of some medicines such as herbal products or biological drugs, inactivation in gastric pH, and enzymatic degradation reduce the bioavailability of drugs used in NAFLD. NPs offer the possibility of oral administration of many types of medicines despite biological barriers. Improved oral bioavailability was associated with increased water solubility, higher release rate, protecting against enzymatic degradation, improved absorption, and increased mean residence time in the GI tract. In addition, targeted NPs improve absorption via clathrin-mediated endocytosis [122].

The lack of in vitro models that can predict the fate of NPs in the GI tract and evaluate the bioavailability of encapsulated drugs is another issue in research experiments. Current models are based on transwell systems that are easy, inexpensive, and useful, but they cannot accurately simulate the GI environment. In addition, because of the possibility of surface changes and ligand damage, the oral route is not the appropriate way to administrate the most active targeted NPs.

## 2. Conclusion

Because of a significant increase in the prevalence of NAFLD, resulting in liver transplantation and deaths, more effective strategies need to be explored to treat NAFLD and prevent disease progression. The use of NPs as drug carriers is a promising way of making drugs safer and more efficacious. This review has discussed various NP delivery systems that are investigated for the treatment of NAFLD. The development of these delivery systems offers tremendous opportunities for the management of liver diseases such as NAFLD. We show that employing NPs as drug carriers has enormous potential to improve the bioavailability of therapeutic agents in NAFLD treatment. In Table 1, the types of nanoparticles reviewed in the previous sections have been classified and linked to related bibliographic sources. Given recent progress acquired from laboratory studies, more nanoparticle-based delivery platforms will be employed in the therapeutic field of liver diseases. However, the large-scale production of nanoparticles is still a daunting process. Fortunately, advances in large-scale production continue to facilitate the clinical application of nanoparticle delivery systems. In particular, we envisage that more nanoplatforms will be employed to overcome barriers in the oral delivery of drugs in managing metabolic diseases such as NAFLD.

## Figures and Tables

**Figure 1:** Multiple parallel hits hypothesis in nonalcoholic fatty liver disease (reproduced with permission from [11]).

**Figure 2:** Liver anatomy. (a) Entire organ, (b) blood supply, and (c) schematic of cells, ducts, and blood vessels based on the research article [123].

**Figure 3:** Receptors or cellular targets on liver cells for nanoparticles active targeting to the liver. (a) Hepatocyte, (b) hepatocellular carcinoma cell, (c) hepatic stellate cells (HSC), (d) Kupffer cell, and (e) endothelial cells (reproduced from [15] with permission from the Royal Society of Chemistry).

**Table 1:** Nanoformulation approaches designed to improve treatment efficiency in NAFLD.

Nanoparticle	Advantages		Payload	References
Nanoemulsion	Simple preparation method, transparent, stable over the time		Pumpkin seed oil, vitamin D, cuminaldehyde, silymarin, carotenoid	[25, 30, 32, 36, 37, 39, 43]

Liposome	FDA-approved, biocompatibility, biodegradability, the ability to carry a large payload		Fenofibrate, biacalin, deoxyschizandrin, eicosapentaenoic acid (EPA), docosahexaenoic acid (DHA), curcumin	[48, 49, 54, 57, 66]

Self-emulsifying drug delivery systems (SEDDS)	Improve oral bioavailability of poorly water-soluble drugs		Silymarin, silybin	[68, 70, 71]

Micelles	Excellent stability, reproducible scale-up, wide drug loading range		Xanthohumol, SKLB023, resveratrol	[77, 78, 87]

Polymeric nanoparticle	FDA-approved, biocompatibility, versatility		Curcumin, resveratrol, rapamycin, fenofibrate, bisindolylmaleimide I (BIM-I), siRNA	[91–93, 96, 99, 100]

Nanogel	Biocompatibility, controlled release systems		Hydroxytyrosol (HT)	[102]

Other nanoparticles	Cerium oxide nanoparticles (CeO2NPs)	Hepatoprotective effect	siRNA, gene delivery, curcumin	[104, 109, 116, 120]
	Zinc oxide nanoparticles (ZnO-NPs)	Induction of apoptosis in macrophages		
	Biguanide incorporated chitosan particles	Gene transfection efficiency, exert similarly biological activity as metformin		
	Albumin-based nanoparticle	Biodegradability, nontoxicity, nonimmunogenicity		

## Data Availability

There are no raw data associated with this review article.
